# Identification of novel genes in aging osteoblasts using next-generation sequencing and bioinformatics

**DOI:** 10.18632/oncotarget.22748

**Published:** 2017-11-28

**Authors:** Yi-Jen Chen, Wei-An Chang, Ming-Shyan Huang, Chia-Hsin Chen, Kuan-Yuan Wang, Ya-Ling Hsu, Po-Lin Kuo

**Affiliations:** ^1^ Graduate Institute of Clinical Medicine, College of Medicine, Kaohsiung Medical University, Kaohsiung, Taiwan; ^2^ Department of Physical Medicine and Rehabilitation, Kaohsiung Medical University Hospital, Kaohsiung, Taiwan; ^3^ Division of Pulmonary and Critical Care Medicine, Kaohsiung Medical University Hospital, Kaohsiung, Taiwan; ^4^ Department of Internal Medicine, E-DA Cancer Hospital, Kaohsiung, Taiwan; ^5^ School of Medicine, I-Shou University, Kaohsiung, Taiwan; ^6^ Department of Physical Medicine and Rehabilitation, School of Medicine, Kaohsiung Medical University, Kaohsiung, Taiwan; ^7^ Division of Geriatrics and Gerontology, Kaohsiung Medical University Hospital, Kaohsiung, Taiwan; ^8^ Graduate Institute of Medicine, College of Medicine, Kaohsiung Medical University, Kaohsiung, Taiwan; ^9^ Institute of Medical Science and Technology, National Sun Yat-Sen University, Kaohsiung, Taiwan

**Keywords:** aging osteoblasts, next-generation sequencing, bioinformatics, microRNA, messenger RNA

## Abstract

During the aging process, impaired osteoblastic function is one key factor of imbalanced bone formation and age-related bone loss. The aim of this study is to explore the differentially expressed genes in normal and aged osteoblasts and to identify genes potentially involved in age-related alteration in bone physiology. Based on next generation sequencing and bioinformatics analysis, 12 differentially expressed microRNAs and 22 differentially expressed genes were identified. Up-regulation of miR-204-5p was validated in an array of osteoporotic hip fracture in the Gene Expression Omnibus database (GSE74209). The putative targets for miR-204-5p were Kruppel-like factor 7 (*KLF7*) and SRY-box 11 (*SOX11*). Ingenuity Pathway Analysis identified *SOX11*, involved in osteoarthritis pathway and differentiation of osteoblasts, together with miR-204-5p, a potential upstream regulator, suggesting the critical role of miR-204-5p-*SOX11* regulation in the aging process of human bones. In addition, as semaphorin 3A (*SEMA3A*) and ephrin type-A receptor 5 (*EPHA5*) were involved in nervous system related biological functions, we postulated a potential linkage between *SEMA3A*, *EPHA5* and development of neurogenic heterotopic ossification. Our findings implicate new candidate genes in the diagnosis of geriatric musculoskeletal disorders, and provide novel insights that may contribute to the elaboration of new biomarkers for neurogenic heterotopic ossification.

## INTRODUCTION

Life expectancy has increased during the past decades, and issues related to global aging are growing. At present, the average percentage of elderly around the world is about 15%, and this number is expected to increase to approximately 20% by 2050 [1]. With aging, body systems and organs undergo physiological changes, resulting in increased comorbidities [2].

Bone structure consists of trabecular bone and cortical bone. Trabecular bone is more metabolically active and its bone mineral density begins to decrease in young adulthood. Cortical bone provides mainly structural support, and its bone mineral density remains stable until middle age and then begins to decrease [3]. Post-menopausal increase in bone turnover and bone porosity is the primary factor for women having more overall cortical bone loss than men throughout life [4]. The maintenance of bone health relies on the balanced remodeling of osteoblasts and osteoclasts. Osteoblasts are responsible for bone formation, whereas osteoclasts are responsible for bone resorption [5]. Disequilibrium of osteoblast and osteoclast activities related to aging, metabolic diseases and hormonal changes may lead to bone fragility and clinical disorders such as osteoporosis [6].

MicroRNAs are small non-coding RNAs of 20–22 nucleotides which regulate gene expressions through a post-transcriptional manner, acting as key regulators in various biological processes [7]. Novel targets in many biological functions and human diseases have been discovered by microRNA profiling, including bone remodeling [8, 9] and osteoarthritis (OA) [10, 11]. Dysregulated microRNAs were also identified as affecting the differentiation and proliferation of multipotent mesenchymal stem cells (MSCs), thereby regulating bone formation [12–14]. In the era of an aging population, research on the aging processes of different organ systems using microarray and next generation sequencing (NGS) approaches has also evolved [15–17]. NGS technique provides high-throughput genomic profiling of the whole genome, including DNA, RNA and small RNA sequencing, and DNA methylation [18]. The differentially expressed profiling results obtained from NGS require further analysis using bioinformatics approaches to identify candidate genes and/or microRNAs of interest. In this study, we sought to identify potential microRNA-mRNA interactions in aged osteoblasts using different bioinformatics databases and tools, including Ingenuity^®^ Pathway Analysis (IPA), Database for Annotation, Visualization and Integrated Discovery (DAVID) [19], Gene Expression Omnibus (GEO) [20], and miRmap [21].

Both OA and osteoporosis are common age-related musculoskeletal disorders. Currently, the diagnosis of OA and osteoporosis relies largely on imaging studies, and disease severity does not necessarily correlate with clinical symptoms. The aim of this study is to explore the differentially expressed genes in aged osteoblasts and to identify potential genes involved in age-related alterations in bone physiology. Through the NGS and bioinformatics approaches, we hope to provide novel perspectives in the future development of biomarkers in advancing diagnosis and evaluation of therapeutic efficacy of age-related bone diseases among the geriatric population.

## RESULTS

### Confirmation of cell senescence of osteoblasts at late passages

The cellular aging of human osteoblasts, like many other cell types, demonstrated characteristic morphological changes and increased proportion of cells with positive β-galactosidase staining [22]. We observed the serial morphological changes of human osteoblasts of different passages. As the osteoblasts were cultured to later passages, the cell morphologies changed from thin, spindle shape to flattened, irregular shape with increased intracellular debris (Figure 1A). The proportion of β-galactosidase positive cells also increased in the later passages, as shown in Figure 1B, indicating the osteoblast senescence.

**Figure 1:** Morphological changes and β-galactosidase staining of human primary osteoblasts of different passages confirmed the osteoblast senescence at later passages The morphological changes (**A**) and β-galactosidase staining (**B**) of human primary osteoblasts of second, fourth, and seventh passages were identified. The morphologies of young osteoblasts were thin and spindle-shaped. Increased number of cells with flattened and irregularly-shaped morphologies and increased intracellular debris were observed at later passages (arrow). The cells with blue staining indicated β-galactosidase-positive cells (arrow), representing senescent cells. The cells were observed under light microscope at 10X field.

### Identification of potential microRNA-mRNA interactions in aging osteoblasts

Studies have indicated the importance of microRNA regulation on the gene expression in the aging process of human musculoskeletal system [23–25]. To study the microRNAs potentially involved in the aging process of osteoblasts, the NGS results of small RNA-seq from human primary osteoblasts of first (P1) and eighth (P8) passages were obtained. MicroRNAs with > 2.0-fold differential expression and reads per million (RPM) > 10 were selected. Twenty-nine microRNAs were identified, as listed in Table 1. To identify potential microRNA-mRNA interactions in aging osteoblasts, we first analyzed the putative targets of 10 up-regulated microRNAs and 19 down-regulated microRNAs from NGS results using miRmap microRNA putative target predictor, and selected targets with miRmap scores > 99.0 that indicated high predictive strength of repression. A total of 381 target genes (412 potential interactions) predicted by 10 up-regulated microRNAs, and 606 genes (790 potential interactions) predicted by 19 down-regulated microRNAs were identified. We then matched the selected target genes to our RNA-seq with > 2.0 fold down- or up-regulated mRNAs, using the “Compare Dataset” tool in the IPA. Matched results identified 22 target genes (11 down-regulated genes and 11 up-regulated genes), as shown in Figure 2A. The heatmap analysis of 29 differentially expressed microRNAs with z-score values was shown in Figure 2B.

**Table 1:** Differentially expressed microRNAs identified from P1 and P8 osteoblasts

miRNA name	precursor	OB-P8 seq (norm)	OB-P1 seq (norm)	Fold Change OB-P8/OB-P1	Direction of Change
hsa-miR-376a-5p	hsa-mir-376a-1	94.85	19.73	4.81	Up
hsa-miR-204-5p	hsa-mir-204	294.77	64.6	4.56	Up
hsa-miR-136-5p	hsa-mir-136	143.84	41.23	3.49	Up
hsa-miR-137	hsa-mir-137	37.94	12.13	3.13	Up
hsa-miR-132-3p	hsa-mir-132	207.12	67.07	3.09	Up
hsa-miR-181c-5p	hsa-mir-181c	224.29	77.33	2.90	Up
hsa-miR-193a-3p	hsa-mir-193a	122.83	43.4	2.83	Up
hsa-miR-4792	hsa-mir-4792	57.39	23.87	2.40	Up
hsa-miR-497-5p	hsa-mir-497	72.28	33.14	2.18	Up
hsa-miR-27a-3p	hsa-mir-27a	5256.87	2456.33	2.14	Up
hsa-miR-424-5p	hsa-mir-424	71.56	151.4	-2.12	Down
hsa-miR-708-5p	hsa-mir-708	15.37	32.84	-2.14	Down
hsa-miR-20a-5p	hsa-mir-20a	106.5	227.74	-2.14	Down
hsa-miR-708-3p	hsa-mir-708	16.09	34.82	-2.16	Down
hsa-miR-22-5p	hsa-mir-22	21.61	46.85	-2.17	Down
hsa-miR-222-5p	hsa-mir-222	25.45	55.92	-2.20	Down
hsa-miR-1180-3p	hsa-mir-1180	30.98	68.94	-2.23	Down
hsa-miR-148a-5p	hsa-mir-148a	48.99	109.09	-2.23	Down
hsa-miR-335-5p	hsa-mir-335	589.9	1331.53	-2.26	Down
hsa-miR-138-1-3p	hsa-mir-138-1	12.37	31.56	-2.55	Down
hsa-miR-1260b	hsa-mir-1260b	359.61	932.17	-2.59	Down
hsa-miR-1260a	hsa-mir-1260a	321.06	841.03	-2.62	Down
hsa-miR-424-3p	hsa-mir-424	39.98	120.63	-3.02	Down
hsa-miR-452-5p	hsa-mir-452	38.78	122.5	-3.16	Down
hsa-miR-224-5p	hsa-mir-224	113.59	373.32	-3.29	Down
hsa-miR-378a-3p	hsa-mir-378a	121.39	444.83	-3.66	Down
hsa-miR-335-3p	hsa-mir-335	791.86	3652.64	-4.61	Down
hsa-miR-146b-3p	hsa-mir-146b	11.29	69.04	-6.12	Down
hsa-miR-146b-5p	hsa-mir-146b	186.47	1794.21	-9.62	Down

**Figure 2:** Identification of differentially expressed microRNAs and genes with potential microRNA-mRNA interactions in human primary osteoblasts (**A**) Next generation sequencing (NGS) analysis identified 504 up-regulated genes and 385 down-regulated genes in human primary osteoblasts of eighth passage (P8), compared to first passage (P1) (> 2.0-fold change), where 399 up-regulated genes and 355 down-regulated genes were mapped using Ingenuity Pathway Analysis (IPA) database. In addition, 10 up-regulated microRNAs and 19 down-regulated microRNAs were selected (> 2.0-fold change and threshold of reads per million (RPM) >10), which predicted 381 and 606 putative targets by miRmap (score≥ 99.0), respectively. Among all identified putative targets, 378 targets predicted by 10 up-regulated microRNAs and 599 targets predicted by 19 down-regulated microRNAs were mapped in IPA database. These selected targets and differentially expressed genes were matched by the “Compare Dataset” tool in the IPA, and revealed 22 potential microRNA-mRNA interactions. ^*^One of the mapped genes was not identified in our NGS dataset. (**B**) The heatmap analysis of differentially expressed microRNAs from P1 and P8 osteoblasts with z-score values were shown.

### Differentially expressed miR-204-5p and miR-335-3p in osteoporotic hip bone

The 5 up-regulated microRNAs and 7 down-regulated microRNAs with corresponding putative targets of aged osteoblasts identified via Venn diagram analysis (11 down-regulated genes and 11 up-regulated genes, respectively) are listed in Table 2. To confirm whether these identified microRNAs are of clinical significance in the aging process of bones, we searched the GEO database for related arrays in age-related bone diseases such as OA and osteoporosis, and found a related array (GEO accession: GSE74209). The array contained bone specimens from six women with osteoporotic femoral neck fractures, and six women with hip OA but no osteoporosis [26]. The 12 differentially expressed microRNAs were individually analyzed with corresponding identifiers from the ID column of the array dataset for expression values. The results showed that miR-204-5p was significantly up-regulated, whereas miR-335-3p was significantly down-regulated, in women with osteoporotic hip fractures compared to those with hip OA but no osteoporosis (Figure 3A and 3B). As listed in Table 2, *KLF7* and *SOX11* were the predicted targets of miR-204-5p, while *KIAA1462* and *SVIP* were targets of miR-335-3p.

**Table 2:** Genes selected between putative targets of microRNA and differentially expressed genes from NGS database

Up-regulated microRNA	Target down-regulated mRNA	Gene name	Fold-change (P8 vs. P1)
hsa-miR-497-5p	*ADAMTS12*	ADAM metallopeptidase with thrombospondin type 1 motif, 12	5.31
	*CD40*	CD40 molecule	4.28
	*COL12A1*	collagen, type XII, alpha 1	3.89
	*SIK1*	salt-inducible kinase 1	3.38
	*PID1*	phosphotyrosine interaction domain containing 1	3.22
	*RAB3IP*	RAB3A interacting protein	5.88
hsa-miR-193a-3p	*AJUBA*	ajuba LIM protein	3.38
	*NT5DC3*	5′-nucleotidase domain containing 3	2.85
hsa-miR-204-5p	*KLF7*	Kruppel-like factor 7	2.02
	*SOX11*	SRY (sex determining region Y)-box 11	6.97
hsa-miR-181c-5p	*RAB3IP*	RAB3A interacting protein	5.88
hsa-miR-27a-3p	*SLC7A11*	solute carrier family 7 member 11	2.55
**Down-regulated microRNA**	**Target up-regulated mRNA**	**Gene name**	**Fold-change (P8 vs. P1)**
hsa-miR-1260a	*CACNB4*	calcium channel, voltage-dependent, beta 4 subunit	9.51
hsa-miR-1260b	*CACNB4*	calcium channel, voltage-dependent, beta 4 subunit	9.51
hsa-miR-20a-5p	*CELF2*	CUGBP Elav-like family member 2	5.90
	*EPHA5*	ephrin type-A receptor 5	20.28
	*FGD4*	FYVE, RhoGEF and PH domain containing 4	2.50
hsa-miR-424-5p	*E2F7*	E2F transcription factor 7	2.10
	*PDK4*	pyruvate dehydrogenase kinase, isozyme 4	8.54
	*PLAG1*	pleiomorphic adenoma gene 1	2.65
	*SEMA3A*	semaphorin 3A	9.58
hsa-miR-335-3p	*KIAA1462*	KIAA1462	2.12
	*SVIP*	small VCP interacting protein	2.74
hsa-miR-335-5p	*KIAA1462*	KIAA1462	2.12
hsa-miR-224-5p	*MOXD1*	monooxygenase DBH-like 1	3.28

**Figure 3:** Analysis of 12 microRNAs with potential interactions in the GEO database The 5 up-regulated microRNAs (**A**) and 7 down-regulated microRNAs (**B**) were validated in a related array (GSE74209) from the GEO database. Significant upregulation of miR-204-5p and downregulation of miR-335-3p were observed in women with osteoporotic hip fractures, when compared to those with hip osteoarthritis without osteoporosis. ^*^ indicated *p* < 0.05, and n.s. indicated no statistical significance. (ID reference: miR-497-5p, 2829; miR-193a-3p, 2567; miR-204-5p, 2564; miR-181c-5p, 861; miR-27a-3p, 845; miR-1260a, 411; miR-1260b, 382; miR-20a-5p, 4278; miR-424-5p, 587; miR-335-3p, 321; miR-335-5p, 1996; miR-224-5p, 2367).

We further sought to identify diseases and functions associated with the 22 target genes analyzed using IPA software. Three networks associated with cancer, organ injury and abnormality, tissue morphology, endocrine system disorders, cellular development, cell-mediated immune response and cellular movement were identified, with networks 1 and 2 having higher scores and 10 focused molecules (Table 3). Matched to the putative targets analyzed in the previous section, three of the four predicted targets (*KLF7*, *SOX11* and *SVIP*) were involved in network 2 (Figure 4A). Of the two microRNAs identified, miR-204-5p was one of the upstream regulators (*p*-value of overlap = 8.15E-03, targeting *EPHA5*, *PID1*, *PLAG1* and *SOX11* in this dataset) identified in the IPA analysis result (Figure 4B). Using the overlay tool, we identified the molecules involved in the osteoarthritis pathway, Wnt/β-catenin pathway, and differentiation of osteoblasts (marked in purple in Figure 4B), with *SOX11* the only molecule simultaneously involved. We then analyzed the binding site and sequence of miR-204-5p in the 3′UTR of *SOX11* in miRmap, TargetScan and miRDB. Three target sites of miR-204-5p on *SOX11* 3′UTR were identified in all of the above microRNA target prediction databases, including the position of 589-595 (miRmap score 99.41), 985–991 (miRmap score 96.12) and 5910–5916 (miRmap score 93.40) (Figure 5). The results suggest that the regulation of miR-204-5p on *SOX11* may play a critical role in the aging process of human bone.

**Table 3:** Networks associated with genes targeted by miRNAs differentially expressed in osteoblasts

	Top diseases and functions	Score	Focus molecules	Molecules in network
1	Cancer, organismal injury and abnormalities, tissue morphology	24	10	2′ 5′ oas, Act1, **ADAMTS12, AJUBA**, Akt, **CD40**, CD80/CD86, **CELF2**, Chil3/Chil4, Cr3, EFNA1, **EPHA5**, ERK, ERK1/2, F Actin, Fascin, Fcer, **FGD4**, GTPase, Hla-abc, IGHE, IL6, Jnk, N-Cadherin, **Pde4, PDK4**, PID1, Proinsulin, **RAB3IP**, RET, **SEMA3A**, SEMA3D, sphingomyelinase, TRAF, Traj18
2	Cancer, endocrine system disorders, organismal injury and abnormalities	24	10	Adaptor protein 2, ADSS, ATOH7, BSN, **CACNB1**, CACNB4, CCND1, CGB3, **COL12A1**, DCN, **E2F7**, ELAVL1, Hspg, IER2, IGIP, **KLF7, SIK1**, miR-16-5p, miR-3175, miR-486-3p, MTORC1, N-Cadherin, **NT5DC3, PLAG1**, RARA, RET, **SLC7A11**, SNRK, **SOX11, SVIP**, TGFB1, TMSB15A, VEGFA, VPREB3, WNT3A
3	Cellular development, cell-mediated Immune response, cellular movement	4	2	GLRX3, **KIAA1462**, miR-1249-5p, miR-149-3p, miR-1972, miR-2110, miR-3103-5p, miR-4271, miR-5584-5p, miR-6967-5p, **MOXD1**, SUMO3, TMEM25

**Figure 4:** Prediction of network of genes involved in the regulation of miR-204-5p in aging human osteoblasts (**A**) The 22 candidate genes identified from human osteoblasts were analyzed by IPA for network analysis. The network analysis revealed 10 out of 22 genes involved in a network associated with cancer, endocrine system disorders, organismal injury and abnormalities, and three of the four putative targets (*KLF7*, *SOX11* and *SVIP*) by miR-204-5p and miR-335-3p predictions were involved. Genes colored in green indicated down-regulated expressions, and genes in red indicated up-regulated expressions in our dataset. (**B**) miR-204-5p was analyzed by IPA as a potential upstream regulator in our dataset. Using the overlay tool in IPA, molecules involved in the canonical osteoarthritis pathway, Wnt/β-catenin pathway, and differentiation of osteoblasts were marked in purple, where *SOX11* was the molecule simultaneously involved.

**Figure 5:** The putative binding site of SOX11 for miR-204-5p The target binding site and sequence alignment of miR-204-5p on *SOX11* 3′UTR at positions of 589-595, 985-991 and 5910-5916 were validated in three microRNA target prediction databases, including miRmap (**A**), TargetScan (**B**) and miRDB (**C**).

### Analysis of potential molecules involved in miR-204-5p regulation on *SOX11*

To determine the potential interactions between miR-204-5p-*SOX11* regulation and other downstream effectors in our aging osteoblast database, we identified miR-204-5p as an upstream regulator in IPA results for all differentially expressed genes. The network of miR-204-5p related molecules with overlay tool in the IPA was used, and revealed that *ALPL*, *CYP1B1*, *EGR1*, *GREM1*, *IGFBP5*, *PRDM1* and *SOX11* are associated with differentiation of osteoblast and muscle cells, bone mineralization and mineral density, and osteoclastogenesis (Table 4).

**Table 4:** Potential molecules involved in miR-204-5p regulation on SOX11

Analysis	Function	Molecules
miR-204-5p network	Bone mineral density	ALPL, EGR1, PRDM1
	Differentiation of muscle cells	EGR1, IGFBP5, SOX11
	Differentiation of osteoblast	ALPL, GREM1, IGFBP5, SOX11
	Mineralization of bone	ALPL, GREM1, SOX11
	Osteoclastogenesis	CYP1B1, PRDM1

### Identification of differentially expressed genes in aged human osteoblasts and the potential involved pathways

To further identify pathways involved in the aging process of human bones, we performed RNA-seq by NGS to compare the differentially expressed genes between P1 and P8 human osteoblasts. Differentially expressed genes between P1 and P8 osteoblasts with at least two-fold up-regulation or down-regulation were selected from the NGS data. The NGS results identified 504 up-regulated genes and 385 down-regulated genes in P8, compared to P1 osteoblasts. To determine the potential pathways involved in these differentially expressed genes, the list of these differentially expressed genes was uploaded to IPA for further analysis. IPA analysis revealed 133 significant canonical pathways that were associated with differentially expressed genes of our RNA-seq database. Among the top 10 canonical pathways identified, 30 molecules were involved in OA and rheumatoid arthritis (RA) related pathways (16 up-regulated genes and 14 down-regulated genes in our database). The differentially expressed genes were categorized into 25 networks, where diseases and functions annotation such as bone mineral density, differentiation of osteoblasts, osteoarthritis and damage of cartilage tissue were selected to identify related genes. Network analysis is shown in Figure 6, where *SOX11* was interconnected between the networks of osteoblast differentiation and bone mineral density, and was predicted to inhibit *EGR1* and activate *PRDM1*, two molecules in the bone mineral density network.

**Figure 6:** Merged skeletal diseases and functions network and prediction of target molecules The differentially expressed genes identified in our NGS dataset were analyzed by IPA and categorized into 25 networks, where skeletal diseases and functions annotation, including bone mineral density, differentiation of osteoblasts, osteoarthritis and damage of cartilage tissue were selected to identify related genes. Merged network analysis showed *SOX11* was interconnected between the networks of osteoblast differentiation and bone mineral density, and was predicted to inhibit *EGR1* and activate *PRDM1*, two molecules in the bone mineral density network.

### Upregulation of *EPHA5* and *SEMA3A* involved in the axon guidance pathway

The 22 genes with potential microRNA-mRNA interactions were input into the DAVID database to analyze the related biological processes and pathways, and address potential mechanisms involved in aging osteoblasts. The KEGG pathway analysis in DAVID database was used, and set the cutoff value at EASE=1 to avoid false-negative results in a smaller gene list containing only 22 genes. Result indicated 2 genes, *EPHA5* and *SEMA3A*, were involved in the axon guidance pathway (Table 5). The results were identical to IPA network analysis, where overlay canonical pathway of axon guidance signaling in network 1 from network analysis of these 22 candidate genes revealed the involvement of *EPHA5* and *SEMA3A* (Figure 7). As determined by gene ontology results from functional annotation analysis in DAVID database, the terms of biological processes of the genes of interest are shown in Figure 8. Most of the above-mentioned genes (*KLF7*, *SOX11*, *EPHA5*, and *SEMA3A*) were involved in nervous system related biological functions, including axon guidance, sympathetic nervous system development and dendrite morphogenesis.

**Table 5:** KEGG pathway analysis of 22 candidate genes with potential microRNA-mRNA interactions

Term	Count	Genes	*P*-value	Fold Enrichment
Axon guidance	2	*EPHA5* ↑ *SEMA3A* ↑	1D.2E-1	13.6

EASE = 1.0.

**Figure 7:** Network of genes potentially involved in axon guidance signaling pathway in aging human osteoblasts Overlay canonical pathway of axon guidance signaling in network 1 from network analysis of the 22 candidate genes validated the prediction of *EPHA5* and *SEMA3A* involvement in axon guidance pathway from KEGG pathway analysis.

**Figure 8:** Biological process analysis of candidate genes in aging human osteoblasts Functional annotation analysis of the 22 candidate genes by the DAVID database identified nine terms of biological processes involved. Four genes (*KLF7*, *SOX11*, *EPHA5*, and *SEMA3A*) were involved in axon guidance, sympathetic nervous system development and dendrite morphogenesis. The selected criteria for functional annotation analysis were EASE = 0.1 and fold enrichment > 1.3.

## DISCUSSION

Bone structure consists of trabecular bone and cortical bone. Osteoblasts are distributed in the inner layer of the periosteum and along the trabeculae. They are derived from MSCs, and differentiate into osteocytes [27]. During the aging process, impaired osteoblastic function is the consequence of decreased proliferation and differentiation, and increased cellular senescence of MSCs, leading to imbalanced bone formation and age-related bone loss [3, 28].

Our current study, based on NGS and bioinformatic analysis, identified 22 differentially expressed genes and 12 differentially expressed microRNAs potentially involved in aging osteoblasts. We further analyzed the 12 microRNAs in the GEO database of osteoporotic fracture array data (GSE74209), and found miR-204-5p to be up-regulated in osteoporotic fracture bone, which was also a potential upstream regulator of the 22 candidate genes in aging osteoblasts identified in IPA analysis. The putative target genes for miR-204-5p in our database were identified as *KLF7* and *SOX11*, with *SOX11* the gene of interest. Here, we proposed a novel finding of miR-204-5p-*SOX11* regulation during the process of geriatric musculoskeletal physiological changes.

MiR-204-5p has been reported to be a tumor suppressor microRNA in different cancer types [29–31]. Huang et al. demonstrated that miR-204 inhibited osteogenesis and promoted adipogenesis of bone marrow stem cells through negative regulation of Runx2, an important transcription factor for chondrogenesis and osteogenesis [32]. In a rat model of osteoporosis, miR-204-5p was one of the microRNAs associated with bone metabolism in bone marrow osteoblastic cells [33]. In our current study, we found that miR-204-5p was 4.56-fold up-regulated in aged osteoblasts, which was validated in a GEO array of trabecular bone specimens from osteoporotic hip fractures in elderly women [26]. The results indicate that miR-204-5p may be a key regulator of altered bone health in geriatric population.

*SOX11* is one of the *SOXC* transcription factors comprised of *SOX4*, *SOX11* and *SOX12*. SOXC proteins are expressed in various types of progenitor cells, and potentiate cell survival and differentiation related pathways, regulating prenatal structural development [34, 35]. Deletion of *Sox11* in mice results in reduced ossification and skeletal malformations in multiple sites, suggesting the regulatory role of *SOX11* in enhancing osteoblast differentiation [36, 37]. In a mouse OA model performed by Kan et al., the expression of *Sox11* in the degraded cartilage of the medial knee joint was significantly decreased 4 weeks after OA induction, compared to the lateral side or sham-operated knee joint [38]. Xu et al. also proved promotion of ectopic bone formation in *Sox11*-overexpressed MSCs *in vivo*, and fracture healing in rats [39]. To date, only a few studies have reported the dysregulation of *SOX11* in human musculoskeletal diseases. It was proposed that deletion or point mutation of *SOX11* may be associated with Coffin-Siris syndrome, a congenital neurodevelopmental disorder, which results in cranial and skeletal malformations [40]. Kan et al. investigated 10 human cartilage samples obtained during total knee arthroplasty, which revealed graded decreases in SOX11 protein expression in more severely degraded human articular cartilages [38]. In our study, we proposed the role of miR-204-5p-*SOX11* regulation in aging osteoblasts, and the potential downstream regulation of BMPR1A/Runx2 signaling by *SOX11* (Figure 4B), a signaling pathway involved in osteoporosis and OA [41, 42]. Evidence suggests that *SOX11* not only serves as a key transcriptional factor in embryonic development of the skeletal system, but also take part in maintaining joint homeostasis and the bone healing process. Together, the evidence provides novel insights into investigating the physiological and pathological geriatric changes of the musculoskeletal system.

Using IPA analysis, we identified 10 out of 22 candidate genes from aged osteoblasts to be grouped into one network, where cyclin D1 (*CCND1*) served as a connecting hub (Figure 4A). *CCND1* regulates transition of cell cycle from G1 phase to S phase and tumorigenesis through increased cell proliferation [43]. Cellular senescence has been proposed to be involved in the pathogenesis of OA and age-related bone loss [44]. MiR-204-5p overexpression has been found to induce downregulation of *CCND1*, resulting in differentiation of human MSCs toward adipogenic rather than osteogenic lineage [45]. Zhu et al. also found grade-dependent decrease in mRNA and protein expressions of *CCND1* among the knee OA population, compared to healthy controls [46]. These findings supported our results regarding miR-204-5p regulation in aging bone process, where up-regulated miR-204-5p was postulated to down-regulate *SOX11* and be involved in the cell cycle arrest of osteoblasts, leading to clinical observations of increased bone loss among the geriatric population.

The bioinformatics approach in our study suggests that differentially expressed *SEMA3A* and *EPHA5* in long-term passaged osteoblasts may be associated with biological functions of axon guidance, sympathetic nervous system development and dendrite morphogenesis. This information provides insight into the potential clinical relevance and connection between aging bone and molecular mechanisms of neurogenic heterotopic ossification (HO), a feature of mature bone formation in soft tissue after central nervous system (CNS) injuries like brain and spinal cord [47, 48]. The etiology of HO still lacks consensus, with bone morphogenetic protein (*BMP*) being the most widely proposed molecule involved in the mechanism of HO. Salisbury and colleagues proposed the contribution of neuroinflammation to the migration of osteogenic cells from endoneurial progenitors, and further HO formation in mouse quadriceps muscle [49, 50]. In addition, neuroinflammation promotes increased permeability of blood-nerve-barrier, which facilitates progenitor cell penetration [51]. These findings suggest evidence of interconnection between bone formation and sensory innervation, and may provide a clinical explanation of HO formation in traumatic CNS injuries.

*EPHA5* belongs to the receptor tyrosine kinase family. Studies have suggested *EPHA5* as a candidate inhibitor in the osteogenic differentiation capability of long-term passaged human bone marrow stromal cells [52, 53]. Although up-regulated *EPHA5* in our NGS database of P8 osteoblasts was observed, the association between *EPHA5* and other bone diseases or human aging has not been reported.

SEMA3A, a secreted glycoprotein, is known as one of the axon guidance molecules, participating in the development of central and peripheral nervous systems, and impeding axonal regeneration and repair after injury [54–57]. Recently, the role of *SEMA3A* in bone homeostasis has been explicated, and the balance between sensory input and sympathetic output may modulate bone remodeling [54, 58–60]. SEMA3A acts as an autocrine to regulate neuronal development and osteoblastogenesis, and exerts different regulatory effects in various disease entities [58, 61, 62]. The regulation of *SEMA3A* on bone remodeling was speculated to act through sensory innervation [63]. One study investigated the association between *SEMA3A*, traumatic brain injury and osteogenesis and proposed the role of *SEMA3A* in facilitating fracture healing in traumatic brain injury [64]. However, there is not much literature reporting the association between *SEMA3A* sensory innervation of bone and formation of neurogenic HO. Since early inflammatory signs of HO usually mimic other clinical conditions such as thrombophlebitis and cellulitis, and the maturation of HO formation varies among patients with CNS injury, our current findings provide novel insight in studying the role of *SEMA3A* as a biomarker in the early diagnosis and evaluation of maturation and treatment efficacy of neurogenic HO, and merit further comprehensive investigation.

In conclusion, our study shows that miR-204-5p-*SOX11* regulation plays an important role in the homeostasis of bone in aging osteoblasts, and *SEMA3A* may exert a potential linkage to the development of neurogenic HO, as summarized in Figure 9. Our findings suggest new candidate genes in the diagnostic evaluation of geriatric musculoskeletal disorders, and provide novel insights into investigation of potential biomarkers in neurogenic HO.

**Figure 9:** The proposed novel molecular mechanisms of gene regulations involved in aging osteoblasts

## MATERIALS AND METHODS

### Primary cells and simulation of aging osteoblasts

Human primary osteoblasts were purchased from Lonza (Walkersville, MD, USA) and cultured in specified osteoblast growth medium (Lonza, Walkersville, MD, USA) according to the manufacturer’s recommendation. The first passage of primary osteoblasts, delineated as P1, was defined as cells harvested from directly-thawed vials purchased from Lonza under stable growth conditions. To determine the differential expressions of mRNA and microRNA in aging human osteoblasts in our study, the 8th passage of human primary osteoblasts (P8) were harvested for further RNA extraction, which simulated the aging process.

The characteristics of cellular aging at later passages of human osteoblasts were identified by serial observations of the morphological changes using light microscope (Zeiss Primo Vert, Jena, Germany). In addition, cells of different passages were stained for β-galactosidase to confirm the characteristic of osteoblast senescence, using the Senescence β-Galactosidase Staining Kit (Cell Signaling Technology, Danvers, MA, USA), following the instructions provided by the manufacturer.

### RNA sequencing

The expression profiles of mRNA and microRNA were performed with NGS. Total RNA from harvested cells was extracted by Trizol^®^ Reagent (Invitrogen, USA) according to the manufacturer’s instructions. The quality of extracted RNA was analyzed by OD260 detection using an ND-1000 spectrophotometer (Nanodrop Technology, USA), and samples were readied for further RNA preparation and sequencing analysis of both RNA-seq and small RNA-seq by Welgene Biotechnology Company (Welgene, Taipei, Taiwan). The quality of extracted RNA was confirmed by RNA integrity number (RIN) using Agilent Bioanalyzer (Agilent Technology, USA). The criteria for differentially expressed mRNAs were set at a fold change of more than 2.0. The criteria for differentially expressed microRNAs were set at fold change of more than 2 and reads per million (RPM) of more than 10.

### Ingenuity^®^ Pathway Analysis (IPA)

Ingenuity^®^ Pathway Analysis (IPA) software (Ingenuity systems, Redwood City, CA, USA) provides a broad spectrum of scientific reports that enable researchers with quick searching. In addition, IPA also provides powerful analysis, integration and interpretation of big data derived from such as RNA-seq, small RNA-seq, and proteomics.

### DAVID database

The DAVID bioinformatics resources provide high-throughput and an integrated data-mining environment to analyze gene lists derived from gene sequencing experiments. Genes of interest uploaded into the DAVID database can be further classified into clusters of different functional annotations, involved pathways and diseases. The Expression Analysis Systematic Explorer (EASE) score represents modified Fisher’s exact *p*-value in the DAVID database, and is used to screen for genes potentially involved in specific signaling pathways in our gene list. The default cutoff value of EASE score is set at 0.1, and adjustable by the users. The higher cutoff value we set, the lower significance of our gene list in a signaling pathway. On the contrary, the lower cutoff value we set, the higher significance of our gene list in a signaling pathway. Considering the complex biological data mining process, the EASE scores suggest, rather than decide, which genes are potentially involved in the pathway, and users are recommended to make further judgment of the biological relevance [19].

### Gene Expression Omnibus (GEO)

GEO is a database that accepts array and sequence-based data. The GEO tool provides researchers specific gene expression profiles in datasets. The array with accession number GSE74209 was used in this study to verify the microRNAs of interest, which consisted of femoral neck trabecular bones from 6 female osteoarthritic patients without osteoporosis, and 6 females with osteoporotic fractures [26].

### miRmap database

MiRmap is an open-source software library, developed by Vejnar et al., that provides higher microRNA target prediction through comprehensive approaches, including thermodynamic, evolutionary, probabilistic and sequence-based approaches. Using comprehensive features with linear model to predict the repression strength of a specific microRNA, input of a microRNA of interest can lead to a list of putative target genes with respective miRmap scores, which indicated the predictive strength of repression. Putative microRNA target genes with miRmap scores higher than 99.0 were selected for this study [21, 65].

### Statistical analysis

The raw data obtained from GEO database were analyzed to compare the expression values of candidate microRNAs between two groups, using the Mann-Whitney *U* test with IBM SPSS Statistics for Windows, version 19 (IBM Corp., Armonk, NY, USA).
